The article "Effect and Safety of Painless and Conventional Endoscopic Management of Denture Impaction in the Esophagus" was published in 2022. Journal: Comput Intell Neurosci.

# Effect and Safety of Painless and Conventional Endoscopic Management of Denture Impaction in the Esophagus

**DOI:** 10.1155/2022/9949875

**Published:** 2022-09-26

**Authors:** Li li Tian

**Affiliations:** Second Hospital of Shanxi Medical University, Digestive Endoscopy Center, Taiyuan 030001, Shanxi Province, China

## Abstract

**Objective:**

To improve the level of clinical diagnosis and treatment, reduce the incidence of complications, and provide the basis for clinicians to choose an appropriate treatment, this research explores the removal methods of the impacted denture in the esophagus by endoscopy.

**Methods:**

Based on the clinical information, treatment methods and complications of 72 patients with denture impaction in the esophagus admitted to our hospital from January 2016 to March 2021, which were divided into the group treated with painless endoscopy and the group treated with conventional endoscopy, retrospective analysis of the therapeutic effect and complications was conducted.

**Results:**

There was no statistically significant difference between the two groups in terms of denture removal rate (*P* > 0.05). There were statistically significant differences between the two groups in terms of operating time and incidence rates of complications during and after the procedure. The operating time of the group treated with painless endoscopy was significantly shorter than the group treated with conventional endoscopy (*P* < 0.05). The incidence rates of complications during and after the procedure of the group treated with painless endoscopy were significantly lower than the group treated with conventional endoscopy (*P* < 0.05).

**Conclusions:**

Compared with the conventional endoscopy, painless endoscopic management of denture impaction in the esophagus under general anesthesia with tracheal intubation improves the clinical efficacy and reduces the adverse reactions. Thus, it is worthy of clinical popularization and application.

## 1. Introduction

The upper digestive tract foreign body refers to the upper digestive tract that can not be digested and can not be discharged from the body. Once the upper gastrointestinal foreign body is diagnosed, the size, shape, type, quantity, and location of the foreign body should be known in time to formulate a treatment plan. At present, the common treatment methods for the gastrointestinal foreign body include natural discharge, endoscopic therapy, and surgery [1]. From the published literature, it can be seen that the patients with gastrointestinal foreign bodies in China are mainly treated with sharp foreign bodies such as date pit, bone, and denture. Due to the different types of upper gastrointestinal foreign body, the clinical symptoms and harmfulness are also different [2]. An upper gastrointestinal foreign body is a common digestive emergency in China, requiring emergency treatment. If not handled in time, patients may suffer from complications such as fullness, clonic pain, pyloric obstruction, and even death [3, 4]. In China, 70%–75% of upper gastrointestinal foreign bodies are trapped in the esophagus, with the esophageal inlet being the most common [3, 5]. With the improvement in living standard, the utilization rate of the denture in elderly patients in China is high, and denture has become a common upper digestive tract foreign body. Because the sharp denture with metal clasps at both ends is easily immobilized in the alimentary canal wall and cannot be discharged from the body by itself, it is difficult to remove. If not removed in time, it may lead to massive bleeding, perforation, infection, and damage to adjacent organs, and even endanger life in serious cases. Therefore, it is particularly important for the timely treatment of esophageal immobilized dentures. Emergency gastroscopy for the treatment of the upper gastrointestinal foreign body is a method with high safety and success rate [5, 6], including ordinary gastroscopy and painless gastroscopy. If the sharp object is incarcerated in the esophagus, the impaction of the food ball may cause high obstruction, which requires urgent endoscopic treatment. Compared with surgical operation, endoscopic foreign body removal has the advantages of less trauma, lower cost, and relatively simple operation, which has become the most important means for the treatment of the esophageal foreign body. However, in clinical practice, patients are often reluctant to cooperate in the removal of esophageal foreign bodies under local anesthesia because of fear. Moreover, if the surface local anesthesia is not sufficient, it may cause severe vomiting and struggle, head and neck twisting, and even sitting up, especially for patients with a short neck, mental tension, cervical diseases, and foreign bodies that are difficult to deal with. In these cases, when the gastroscope enters the closed esophageal entrance, it is difficult to see the relationship between the foreign body and the esophagus. If the operation is performed blindly, especially when the forceps are used to remove sharp foreign bodies, such as dentures and nails, because the foreign bodies are often pierced into the esophagus wall, the patient may experience muscle tension. If the doctor's operation is rough, forced clip out, complications will increase significantly. Mild cases of esophageal mucosal injury, bleeding, esophageal perforation and surrounding tissue infection, mediastinal abscess, and other complications, severe cases can injure the aorta, the formation of esophageal aortic fistula, the occurrence of massive bleeding and death. The general anesthesia operation does not involve the patient's cooperation problem. The nondepolarizing agent used can the maximum limit to remove esophageal muscle cramps or lower esophageal muscle tension, especially in the ring at the top of the esophagus pharyngeal constrictor flabby muscle, swallow, reduces the gastroscope to the operation field and friction resistance, promotes the insertion of a gastroscope, thereby reducing bleeding, guarantee the sharpness of the operation field, avoid the blindness of operation, reduce the occurrence of complications, is advantageous to the foreign body removed, And ultimately improve the success rate of surgery.

At present, there are few comparative studies on the safety and effectiveness of ordinary gastroscopy and painless gastroscopy in the treatment of esophageal denture incarceration. This study aims to analyze and compare the treatment success rate and intraoperative and postoperative complications of ordinary gastroscopy and painless gastroscopy in order to provide clinical guidance for the treatment of esophageal denture incarceration.

## 2. Data and Methods

### 2.1. The General Information

The clinical data of 78 patients diagnosed and treated with esophageal denture incarceration in the Second Hospital of Shanxi Medical University from January 2014 to May 2021 were retrospectively analyzed. There were 42 males and 36 females, with a male to female ratio of 1.17 : 1. The average age was (63.9 ± 7.96) years old from 51 to 82 years old, including 28 (35.9%) ≤ 60 years old, 34 (43.6%) from 61 to 70 years old, 15 (19.2%) from 71 to 80 years old, and 1 (1.3%) > 80 years old. 62 cases (79.5%) and 16 cases (20.5%) were diagnosed within 24∼48 hours after onset. 38 patients were treated by endotracheal intubation under general anesthesia, and 40 patients were treated by ordinary gastroscopy outside the class.

### 2.2. Methods

Preoperative preparation: after the patient was admitted to the emergency department of our hospital, detailed medical history was asked, and a chest X-ray examination was performed to determine the location of foreign bodies. For foreign bodies in the middle esophagus, a chest CT examination was required to observe the relationship between foreign bodies and the aorta and heart, and urgent blood routine examination, coagulation, and electrocardiogram examination were performed. Inform the patient's family and sign the consent form. Patients in the class were evaluated by professional anesthesiologists and treated under general anesthesia after endotracheal intubation, while patients outside the class were treated under ordinary gastroscopy.

Operating apparatus: Olympus Q260 endoscopic, Olympus Q290 endoscopic, Rubber cover, transparent cap, foreign body forceps, net basket, and trap.

Procedure: for the ordinary group, local anesthesia was performed in the oropharynx with lidocaine hydrochloride slurry; for the painless group, general anesthesia was performed in the state of tracheal intubation. The endoscope was slowly entered through the left piriform pit with a transparent cap, and the closed esophageal inlet mucosa was removed with the transparent cap to obtain a better operating field [7]. After careful observation, if a denture is found (see Figure 1), carefully explore the position and incarceration of a denture, remove incarceration with foreign body forceps (see Figure 2) and align the long axis of the denture with the axis of the esophagus, place one side of metal clap-ring into the transparent cap, and slowly remove the foreign body. If it is not easy to remove, the denture can be slowly put into the stomach cavity, or if the denture has entered the stomach cavity before treatment, the endoscope should be withdrawn first, and then the rubber sleeve should be put into the stomach cavity with the endoscope. With the aid of foreign body forceps, snare, or net baskets, the denture was loaded into the rubber sleeve (see Figure 3). The foreign body forceps clamped the denture and rubber sleeve, adjusted the direction of the denture to make the long axis of the denture consistent with the long axis of the esophagus, and slowly removed the denture. For the common group of patients, when the denture was taken to the esophagus entrance, the patient was instructed to swallow, the mandible was raised, and the denture was slowly removed. If the denture clings are deeply embedded in the esophageal wall or too large to pass through the esophageal inlet, and the removal fails, the patient will be transferred to surgical treatment.

### 2.3. Observation Indicators

The successful removal rate and operation time of foreign bodies were compared between the two groups, and the occurrence of intraoperative and postoperative complications were observed between the two groups.

### 2.4. Statistical Analysis

SPSS 23 statistical software was used for statistical analysis. All data were in accordance with normal distribution, the mean value of measurement data were expressed as mean ± standard deviation ($\bar{x}$ ± *S*), the comparison between two groups was analyzed by two independent sample *T* test, the counting data were expressed as percentage (%), and the comparison between groups was conducted by *X*^2^ test. *P* < 0.05 was considered statistically significant.

## 3. Results

### 3.1. Comparison of Foreign Body Removal Success Rate and Removal Time between the Ordinary Group and the Painless Group

The success rate of foreign body removal in the painless group was 97.3%, lower than that in the normal group (87.5%), and the difference was not statistically significant (*P* > 0.05). The time of foreign body removal in the painless group was significantly shorter than that in the normal group, and the difference was statistically significant (*P* < 0.05), as shown in Table 1.

### 3.2. The Incidence of Intraoperative and Postoperative Complications in the Normal Group and the Painless Group

In terms of the incidence of total intraoperative and postoperative complications, the painless group was significantly better than the normal group, with statistically significant differences (*P* < 0.05), as shown in Table 2. No serious complications occurred in all patients, similar to previous studies [8]. No major bleeding was observed during the operation. For the small amount of bleeding, the hemostasis can be stopped by ice saline irrigation under endoscopy and endoscopic compression. For local mucous membrane injury, acid suppression, and protection of mucous membrane treatment. For the patients with esophageal perforation, endoscopic placement of the nasojejunal nutrition tube and nasal feeding diet improved significantly.

## 4. Discussion

The denture is a common cause of esophageal foreign body incarceration, which is mostly seen in the elderly [9]. However, due to the X-ray transparency of denture materials, it is often difficult to get a clear diagnosis in time, affecting treatment [10]. Therefore, esophageal denture incarceration is prone to a higher risk of complications, such as esophageal perforation, diverticulum, fistula formation, or intestinal obstruction, which may endanger life. How to treat esophageal denture incarceration in an effective way is of great significance to the life safety of patients.

At present, with the progress of various minimally invasive techniques under gastroscopy, gastroscopy has become the preferred treatment for the removal of upper gastrointestinal foreign bodies [11]. Endoscopic treatment of gastrointestinal foreign body has the advantages of small trauma, high success rate, low risk, and low cost [12, 13]. Studies have shown that emergency endoscopic extraction should be performed actively for dentures incarcerated in the esophagus [14–16]. Removal of an upper gastrointestinal foreign body by ordinary gastroscopy is simple and economical, but it is easy to cause adverse reactions such as nausea and vomiting in patients during the operation [17]. With the rapid development of medical technology, painless gastroscopy has become increasingly mature and widely used in clinical practice. However, there are still little research data on its application in removing incarcerated denture of the esophagus. Exploring the safe and effective extraction method of esophageal incarceration denture under endoscopy can better guide clinicians in choosing the appropriate treatment mode, improve the success rate of surgery and reduce clinical complications.

Observation and analysis of dentures incarcerated in the esophagus treated by emergency endoscopy in our department showed that most of them had sharp reverse multiple metal clasps, which were easily incarcerated in the three strictures of the esophagus, and the first stenosis (esophageal entrance) was more common [18, 19]. Usually, the esophagus entrance is closed and relatively narrow.

However, in the treatment of ordinary gastroscopy, the patient's treatment compliance is poor due to pharyngeal irritation, tension, and fear, and the operator needs to enter the scope several times. The patient's nausea and involuntary defensive actions make the operation more difficult [15, 20, 21]. Zhang et al. [22] study found that propofol intravenous anesthesia raised the success rate of the esophageal foreign body at the same time can shorten the treatment time, avoid taking too much for patients in the process of foreign body reaction mucosal injury, at the same time can also be used for criminals, children and mental patients cannot cooperate with the special groups, such as expanded gastroscope treatment indications. The painless method is general anesthesia under tracheal intubation, which can not only put the patient in an unconscious state but also relax the esophageal muscle of the patient. Muscle relaxation drugs cause the muscles at the entrance of the esophagus to be in a relaxed state, which relaxes the most easily incarcerated foreign bodies and reduces the operation difficulty of removing incarceration and removing foreign bodies [23]. In addition, under tracheal intubation and general anesthesia, the use of muscle relaxants can avoid secondary mucosal damage, and even perforation of the inverted metal clings at the entrance of the esophagus during the removal of partial removable dentures with occluded metal clings in the middle and lower segments of the esophagus and stomach, thus improving the success rate of removal and reducing the incidence of complications. From this retrospective study, we found that there was no statistically significant difference in the success rate of removing dentures between ordinary gastroscopy and painless endotracheal intubation under gastroscopy, suggesting that painless gastroscopy is an effective operation for removing occluded dentures. In terms of operation time and intraoperative complications, compared with the ordinary group, painless treatment with endotracheal intubation has obvious advantages, suggesting that painless gastroscopic removal of esophageal impingement denture is relatively safe and conducive to the smooth development of the treatment process. In addition, compared with ordinary gastroscopy, painless gastroscopy has fewer postoperative complications, suggesting that painless gastroscopy is relatively safe. Therefore, this study concluded that painless gastroscopy is a safe, effective, and ideal means for the treatment of esophageal incarceration dentures, with obvious overall advantages and worthy of widespread promotion and application in clinical practice.

Current problems that need to be improved: tools for foreign body removal: various applicable instruments that need to be developed because of the variety of foreign body types and shapes. ② Gastroscopy also has its own limitations: in cases where the foreign body is small, stays for a long time, and the surrounding hematoma is formed, it is more difficult to clamp the foreign body because it does not show well. For patients with both ends of the foreign body inserted into the anterior and posterior walls of the esophagus, do not rush to clamp the foreign body after discovery. The operation should be cautious and careful, do not take it roughly and forcibly. Otherwise, it may cause perforation, and avoid surgery as much as possible. ③ When withdrawing the foreign body and gastroscope together, be sure to confirm whether the foreign body clamp grasps the foreign body firmly to avoid dropping the foreign body in the epiglottis when withdrawing or even aspirating to the trachea by mistake. If not handled properly, the consequences of accidental aspiration to the trachea are severe. ④ If other diseases or perforation risks are associated, timely hospitalization should be followed by treatment, and relevant departments should fully collaborate in preparing for resuscitation surgery.

## 5. Conclusion

In conclusion, compared with ordinary gastroscopy, painless gastroscopy is recommended for the clinical treatment of incarcerated dentures. Painless gastroscopy has high safety, high patient compliance and comfort, low incidence of adverse reactions, fewer postoperative complications, ideal prognosis, and simple operation. Of course, this study is a retrospective study, and some clinical data, such as the size of a denture and the number of a metal clasp, cannot be accurately counted, which may have a corresponding impact on the results. Therefore, more prospective, multi-center studies are needed to clarify further.

## Figures and Tables

**Figure 1:** Esophageal incarceration denture.

**Figure 2:** Foreign body forceps clamp denture.

**Figure 3:** The denture in the stomach cavity is inside the rubber sheath.

**Table 1:** Comparison of extraction success rate and operation time between ordinary group and painless group.

Groups	Take out the successful (*n*, %)	Take out the failure (*n*, %)	Operating time (min, $\bar{x}$ ± *s*)
Normal group	35 (87.5%)	5 (12.5%)	17.55 ± 1.77
Painless group	37 (97.3%)	1 (2.7%)	15.33 ± 1.93
*χ* ^2^ (*t*)	1.464		5.290
*P*	0.226		0.000

**Table 2:** Comparison of intraoperative and postoperative complications between the normal group and the painless group (*n*, %).

Groups	Mucosal injury	Bleeding	Perforated	Infection	Aspiration	Total
Normal group	8 (20.0%)	2 (5.00%)	3 (7.50%)	1 (2.50%)	2 (5.0%)	16 (40.0%)
Painless group	3 (7.89%)	0 (0%)	1 (2.63%)	0 (0%)	1 (2.63%)	5 (13.15%)
*χ* ^2^	1.464	0.462	0.212	0	0	5.837
*P*	0.226	0.497	0.645	1.000	1.000	0.016

## Data Availability

The datasets generated during and/or analyzed during the current study are available from the author on reasonable request.
